The article "Study on the Effect of Bushen Zhuanggu Tablet Combined with Conventional Regimen on Bone Mineral Density Improvement, Functional Recovery and Fracture Risk Prevention in Patients with Postmenopausal Osteoporosis" was retracted in 2023. Reasons: signs of a paper mill; compromised peer review; unreliable results or conclusions.

# Study on the Effect of Bushen Zhuanggu Tablet Combined with Conventional Regimen on Bone Mineral Density Improvement, Functional Recovery and Fracture Risk Prevention in Patients with Postmenopausal Osteoporosis

**DOI:** 10.1155/2023/4846392

**Published:** 2023-07-07

**Authors:** Tianliang Chen, Guilan Li, Yongtao Xu

**Affiliations:** ^1^The Second Clinical Medical College of Guangzhou University of Chinese Medicine, China; ^2^Department of Orthopedics, Gaozhou Hospital of Traditional Chinese Medicine, China; ^3^Department of Encephalopathy, Gaozhou Hospital of Traditional Chinese Medicine, China

## Abstract

**Objective:**

This case-control study was to explore the effect of Bushen Zhuanggu tablet combined with routine regimen on bone mineral density (BMD) improvement, functional recovery, and fracture prevention in postmenopausal osteoporosis (PMOP) patients.

**Methods:**

180 postmenopausal osteoporosis patients were randomly selected from communities A, B, and C cohorts as research subjects from January to May 2021. The study subjects were divided into three groups. The groups were in a 1 : 1 ratio according to the principles of nonrandomised, concurrent controlled trials, and methods. There were 60 participants in each group (group A, group B, and group C). Group A was treated with Bushen Zhuanggu tablet for antiosteoporosis + basic treatment (calcium supplement and vitamin D). Group C was given Bushen Zhuanggu tablet for antiosteoporosis intervention. Group B was given basic treatment (calcium supplement and vitamin D supplementation) as a control group. The follow-up time was 6 months after treatment. Finally, we compare the differences in calcium and phosphorus metabolism indexes, BMD, bone metabolism indexes, upper and lower limb muscle strength, and quality of life scores.

**Results:**

Group A, B, and C's effective rate was 98.33%, 80.00%, and 93.33%, respectively. The group A's effective rate was significantly higher than that in group B and C, and the difference was statistically significant (*P* < 0.05). After 6 months intervention, the levels of serum Ca^2+^, serum phosphorus (P), serum creatinine (Cr), and parathyroid hormone (PTH) in 3 groups decreased. Ca, P, Scr, and PTH levels in group A were the lowest among study groups, and the difference was statistically significant (*P* < 0.05). The increase in the BMD of lumbar spine, the left femoral neck, and Ward's triangle area of the three groups were observed with the highest data in group A. After 6 months of treatment, the levels of serum N-terminal propeptide of type I procollagen, PINP, and serum osteocalcin (OC) increased, while the levels of *β*-cross-linked C-terminal telopeptide of type I collagen (*β*-CTX) and alkaline phosphatase (ALP) decreased in the three groups. The improvement of all bone metabolic indexes in group A was significantly better than that in B and C groups, and the difference was statistically significant (*P* < 0.05). The enhanced upper limb muscle strength and the shorter standing-walking timing test (TUGT) time were observed after 6 months of treatment. The improvement effect of upper and lower limb muscle strength in group A was significantly better than that in B and C groups, and the difference was statistically significant (*P* < 0.05). There were significant differences in physiological function, life function, general health status, physical pain, mental state, emotional function, vitality, and social function among the three groups after 6 months treatment, and the difference was statistically significant (*P* < 0.05). The score of quality of life in group A was higher than that in B and C groups, and the difference was statistically significant (*P* < 0.05).

**Conclusion:**

Bushen Zhuanggu tablet combined with conventional therapy is effective in the postmenopausal osteoporosis treatment, which effectively increase the BMD, regulate calcium and phosphorus metabolism, promote the recovery of limb function, prevent the recurrence of fracture, and improve the patients' quality of life. This treatment scheme is worth popularizing.

## 1. Introduction

Osteoporosis (OP) has a high incidence in the elderly, especially in postmenopausal women. Osteoporosis is called “silent killer” because of its long incubation period and no obvious symptoms in the early stage. According to statistics, by 2019, the global incidence of osteoporosis has exceeded 200 million, and an average of 20 fractures per minute is caused by osteoporosis [1, 2]. Osteoporosis can occur in all age groups, among which postmenopausal women and elderly men have the highest incidence. Postmenopausal osteoporosis (PMOP), which accounts for the largest proportion, belongs to primary osteoporosis type I [3]. According to the survey, the prevalence rate of osteoporosis in women aged 40-50 in China is 4.3% [4, 5]; women over 50 is 32.1%; women over 65 is 51.6%. The prevalence rate in rural areas is slightly higher comparing with the one in urban areas. Postmenopausal osteoporosis has aroused the public attention and gradually become a significant health issue in our country.

Recent studies have shown that women lose bone mass rapidly during the 5-10 years after menopause with an annual loss rate of about 1.5% to 2.5% [6, 7]. Age, living environment, eating habits, and other diseases and other factors can lead to the occurrence of PMOP. The decline of ovarian function and the decrease of estrogen level are the main reasons. The current antiosteoporosis treatment in Western medicine is based on drugs, supplemented by physiotherapy. Because of its clear mechanism and definite curative effect, drug therapy has become one of the most commonly used drugs in osteoporosis treatment in clinic, mainly including the following categories [8, 9]. Postmenopausal osteoporosis is similar to “bone impotence,” “bone fetish,” “bone withering,” and other diseases in TCM, among which the syndrome of “bone impotence” is the most similar. In TCM theory, the disease is located in the lumbar spine muscles and bones. Its origin lies in the kidney. Generally speaking, the pathogenesis is the deficiency of kidney, liver, and spleen (blood stasis and qi stagnation). The basic drugs include vitamin D and calcium supplements. In addition, bone resorption inhibitors include bisphosphates, calcitonin, estrogen, selective estrogen receptor modulators, and RANKL inhibitors. Bone formation enhancer mainly refers to thyroid hormone analogues. Other mechanism drugs also include active vitamin D and its analogues, vitamin K2 drugs, and strontium salts. The guidelines recommend that when selecting antiosteoporotic drugs in clinic, we should choose broad-spectrum antiosteoporotic drugs such as zoledronic acid, alendronate, and risedronate. However, there are more and more kinds of clinical antiosteoporosis drugs, along with the long-term use of antiosteoporosis drugs and the increase in the number of clinical cases. The continuous emergence of adverse reactions of drugs has also attracted more and more attention. And Western medicine treatment of osteoporosis has a high price, poor tolerance of some patients, adverse reactions and poor long-term efficacy, and other factors, making poor compliance. TCM has relatively few side effects. Basic theories, experimental explorations and clinical studies on the osteoporosis prevention and treatment in Chinese medicine are increasing day by day. Oral drug treatment is the first choice for patients with low BMD but no/low risk of fracture. For those patients with osteoporosis who cannot tolerate oral medication, who have contraindications to oral medication, or who have poor compliance, treatment with injectable, such as zoledronic acid, should be administered once a year [10, 11].

The use of evidence-based and comprehensive treatment can effectively relieve the patients' clinical symptoms. Some scholars have found that the effective components of kidney-tonifying herbs can promote bone formation and inhibit bone resorption. Under normal circumstances, the processes of bone formation are coupled and cooperated with bone resorption. In the case of osteoporosis, bone resorption is greater than bone formation, resulting in bone mass loss. Chinese medicine has unique advantages in the treatment of osteoporosis. However, there are few such scientific studies in clinic, and its application effect remains to be further confirmed [12]. It is necessary to demonstrate the clinical efficacy of TCM therapy in the postmenopausal osteoporosis treatment through scientific research, which can lay a theoretical foundation and thus promote the application of TCM therapy.

## 2. Materials and Methods

### 2.1. General Information

180 randomly selected postmenopausal osteoporosis patients from communities A, B, and C from January to May 2021. Subjects were divided into group A (*n* = 60), group B (*n* = 60), and group C (*n* = 60) in a 1 : 1 ratio according to the measured BMD and the principles and methods of nonrandomised simultaneous controlled trials. Group A was treated with Bushen Zhuanggu tablets for antiosteoporosis + basic treatment (calcium supplementation and vitamin D) for intervention treatment. Group C was treated with Bushen Zhuanggu tablet for antiosteoporosis intervention. Group B was given basic treatment (calcium supplementation and vitamin D supplementation) as the control group. The follow-up time was 6 months after treatment. Group A was aged from 52 to 80 years with an average age of (68.37 ± 7.41) years. Menopause lasted for 1 to 5 years, with average of (2.57 ± 0.51) years. Body mass index (BMI) was 18.76~30.12 kg/m^2^ with average BMI (24.89 ± 2.37) kg/m^2^. Group B was aged from 51 to 79 years, with an average age of (67.34 ± 7.68) years. Menopause lasted from 1 to 6 years with an average of (2.92 ± 0.83) years. BMI ranged from BMI 18.47~29.82 kg/m^2^ with an average BMI of (24.37 ± 2.14) kg/m^2^. Group C was aged from 51 to 79 years, with an average age of (67.34 ± 7.68) years. The time of menopause ranged from 1 to 6 years with the average time of menopause 2.92 ± 0.83 years. The BMI of group C patients was 18.47~29.82 kg/m^2^ and average BMI was 24.37 ± 2.14 kg/m^2^ with *P* value over 0.05, which means there were no significant differences among three groups. This study was approved by the Medical Ethics Council of our hospital. All patients signed the informed consent form for the trial.

Selection criteria is as follows: (1) the selected cases were all diagnosed with postmenopausal osteoporosis, which met the diagnostic criteria in the “Guidelines for Primary Osteoporosis Primary Care (Practical Edition 2019)” formulated in 2011 [13]; (2) the patients had no cognition, language, and intellectual dysfunction, with basic reading and writing skills; (3) all postmenopausal women with *T* value <-2.5; (4) the patients agreed to be followed up for 12 months, who were able to accept and answer telephone follow-up; (5) the patient's clinical data were complete.

Exclusion criteria is as follows: (1) premenopausal osteoporosis (no premenopausal osteoporosis: the patient reported no symptoms related to osteoporosis before menopause, no osteoporosis was found in physical examination, and the BMD test showed that *T* > −1.0. The course of osteoporosis was shorter than the time of menopause); (2) patients with secondary osteoporosis caused by other diseases; (3) those who refused to participate in the trial; (4) those who have recently taken drugs such as glucocorticoids, sex hormones, bisphosphonates, vitamin D, fluoride, and calcium that affect bone metabolism; (5) patients with chronic or severe organ diseases. (6) The individual with severe insufficiency and malignant tumor in either heart, liver, or renal.

### 2.2. Methods

Experimental group A was treated with Bushen Zhuanggu tablet for antiosteoporosis + basic treatment (calcium supplement and vitamin D) for intervention. Group C was given Bushen Zhuanggu tablet for antiosteoporosis for intervention. Group B was given basic treatment (supplemented with calcium and vitamin D) as a control group. Three groups were given health education, including fall prevention and daily life adjustment. Basic treatment content was oral calcium carbonate D3 (Caerqi, Wyeth Pharmaceutical Co., Ltd.) 600 mg/d, active vitamin D (Luo Gaiquan, Roche company) 0.5 *μ*g/d, oral medication for 6 months. Usage of Bushen Zhuanggu tablets is as follows: 3 tablets/time, 3 times/day orally, the drug formula is Bushen Zhuanggu tablets (*Epimedium*, Drynaria, *Rehmannia glutinosa*, *Cornus*, dodder, astragalus, Chinese yam, all angelica, *Panax notoginseng*, danshen, etc.), the prescription has been proved by long-term clinical verification that it has a good effect on improving the clinical symptoms of osteoporosis patients.

### 2.3. Observation Index

#### 2.3.1. Clinical Curative Effect

The therapeutic effects of the three groups were evaluated after treatment, and the specific evaluation criteria were referred to the relevant literature [14]. Markedly, effective was indicated the clinical symptoms of the patient basically disappeared, and the bone mineral density (BMD) level increased by more than 0.05 g cm^2^. Effective was indicated the clinical symptoms of the patient improved, the BMD level increased, but the increase level was lower than 0.05 g cm^2^. Ineffective was indicated the patient's clinical symptoms did not improve or even worsened, and BMD did not increase or decrease. The total effective rate of treatment = (markedly effective + effective) number of cases/total number of cases × 100%.

#### 2.3.2. Muscle Strength Measurement

We carried out the muscle strength measurement before and 6 months after the treatment. The upper limb muscle strength test (two-hand grip strength test): the grip strength test used the electronic grip strength meter (Xiangshan CAMRY, model EH101); the resolution: 0.1KGF; the allowable error: 0.5KGF. Before the test begins, the subject was checked for grip strength disorders. The grip distance was adjusted, and the machine was switched on. The subject held the grip strength meter with the palm of the hand facing inwards and the display facing outwards, with the body upright, feet naturally apart, and arms naturally down, and then grasped as hard as they could. After one practice, the test began. The maximum grip strength of both hands was measured twice, and the average grip strength of two times was taken. After 3 and 6 months of treatment, the standing-walking timing test (TUGT) was performed. The subjects sat on a chair with high 45 cm height, stood up, walked in a straight line of 3 m, and then returned to the seat to sit down. The assessor recorded the time spent on each standing and walking test.

#### 2.3.3. BMD Measurement

BMD was measured before and after treatment. Dual energy X-ray absorptiometry (HOLOGIC, Wi, USA) was used to detect the anterior and posterior lumbar vertebrae (L1 ~ L4), left femoral neck (Neck), and Wards triangle of each subject, expressed by BMD (g/cm^2^). The accuracy of the instrument was 1%, and the repeated measurement error was 1%. In order to reduce the error, all testing operations were completed by the same person. Every day, the instrument was checked with the module provided by the manufacturer, and the test was carried out only after meeting the quality control requirements. The standard for judging bone mass was *T* score: when *T* > −1.0, it meant normal bone mass; when it was (−1.0, −2.5), it meant osteopenia; when *T* < −2.5, it meant osteoporosis [15].

#### 2.3.4. Related Biochemical Indexes of Osteoporosis

The biochemical indexes related to osteoporosis were detected before treatment and 6 months after treatment. (1) Bone metabolic indexes are as follows: procollagen N-terminal propeptide of serum type I (PINP), serum osteocalcin (OC), collagen cross-linked carboxyl terminal peptide type I (*β*-CTX), and alkaline phosphatase (ALP). (2) Calcium and phosphorus metabolic indexes are as follows: serum calcium (Ca2+), serum phosphorus (P), serum creatinine (Cr), and Parathyroid Hormone (PTH).

Fasting peripheral blood 7 ml (including anticoagulant blood vessel 1 ml and procoagulant blood vessel 3 ml) was collected from each subject. The subjects were required to draw elbow venous blood from 8 to 10:00 am with empty stomach. The blood samples were collected on that day by Guangzhou Jinyu testing Technology Co., Ltd. Samples that were not sent on the same day (but ensured that they could be sent on the same day) must be stored in a refrigerator at 4°C within 6 hours. If the sample could not be sent for examination on the same day, the blood collection unit would be responsible for centrifuging and collecting serum (4-5 ml) and freezing it in the refrigerator at −20°C until it was submitted for examination. PINP and *β*-CTX were detected by o-cresolphthalein complex ketone method. OC was detected by radioimmunoassay. ALP and PTH were detected by enzyme-linked immunosorbent assay. Ca^2+^, P, and Cr were detected by RocheCobas8000 biochemical analyzer.

#### 2.3.5. Quality of Life Assessment

The patients' life quality index were recorded before and six months after the intervention. At the same time, the data generated were evaluated by concise health scale (SF-36) [16]. The total score was 100.

#### 2.3.6. Incidence of Refracture

Statistics were made on the number of new fractures in the two groups at 3 months, 6 months, and 12 months after treatment.

### 2.4. Statistical Analysis

SPSS23.0 statistical software was adopted to process the data. The measurement data were presented as ($\bar{x}\pm s$). The group design *T*-test was adopted for the comparison and the analysis of variance was adopted for the comparison between multiple groups. Dunnett's test was adopted for comparison with the control group. The counting data were presented in the number of cases and the percentage, *χ*^2^ test was adopted for comparison between groups, and bilateral test was employed for all statistical tests.

## 3. Results

### 3.1. The Therapeutic Effects among Different Groups

In group A, 36 cases were effective, 23 cases showed effect, and 1 case was ineffective, and the effective rate was 98.33%. The data in group B accordingly was 23, 25, and 12, with the effective rate of 80.0%. The data in group C was 30, 26, and 4, with the effective rate of 93.33%. As a result, the effective rate of group A was significantly higher, and the difference was statistically significant (*P* < 0.05, Figure 1).

### 3.2. Metabolic Indexes of Calcium and Phosphorus

Before treatment, there were no significant differences in the levels of Ca, P, Scr, and PTH in all study groups (*P* > 0.05). After the treatment of 6 months, figure in the 3 groups all decreased. The levels of Ca, P, Scr, and PTH in group A were lower than other groups, and the difference was statistically significant, as showed in Table 1.

### 3.3. Bone Mineral Density Contrast

Before treatment, there were no significant differences in the lumbar anteroposterior BMD, left femoral neck, and Ward's triangle BMD in each group with *P* value over 0.05. After treatment of 6 months, the lumbar spine anteroposterior BMD, left lateral femoral neck, and Ward's triangle BMD were all increased in the three groups, and the difference was statistically significant (*P* < 0.05). All results were shown in Table 2.

### 3.4. Comparison of Bone Metabolic Indexes

Before treatment, there were no significant differences in the levels of PINP, *β*-CTX, ALP, and OC among the three groups (*P* > 0.05). After treatment, the levels of PINP and OC in the three groups increased, while the levels of *β*-CTX and ALP decreased. Compared between groups, the improvement of various bone metabolism indexes in group A was significantly better than that in group B and C, and the difference was statistically significant (*P* < 0.05, Table 3).

### 3.5. Comparison of Upper Limb Muscle Strength and TUGT

Before treatment, there was no significant difference in upper limb muscle strength and TUGT in different study groups (*P* > 0.05). The muscle strength of the upper limbs of the three groups was enhanced, and the TUGT was shortened after treatment. The improvement effect of the muscle strength of the upper limbs and the lower limbs of the group A was significantly better than that of the group B and C, and the difference was statistically significant(*P* < 0.05, Table 4).

### 3.6. Comparison of Quality-of-Life Scores

No significant difference in quality-of-life scores were observed among the three groups before treatment (*P* > 0.05). There were statistical differences in the scores of physiological function, life function, general health status, physical pain, mental state, emotional function, vitality, and social function among the three groups after 6 months of intervention. In addition, the quality of life score of group A was higher than that of group B and C, and the difference was statistically significant (*P* < 0.05, Tables 5 and 6).

### 3.7. Comparison of New Bone Fracture Rate

In group A, the number of new fractures after 3, 6, and 12 months was 0, 1, and 3, respectively. In group B, the number of new fractures after 3, 6, and 12 months was 3, 7, and 14, respectively. The number of new fractures in group C was 2, 5, and 9, respectively, after 3, 6, and 12 months of treatment. The incidence of fracture in group A was lower than that in group B and C at each time point, and the difference was statistically significant (*P* < 0.05, Figure 2).

## 4. Discussion

Osteoporosis (OP) is a common systemic bone disease. OP characterized by decreased bone mass and bone microstructure, Meanwhile, there were increased bone brittleness in the OP patients, which will finally lead to the prone to fracture. The incidence of osteoporosis in the elderly is relatively high. Once a hip fracture occurs, it will directly lead to an increase in disability and mortality in the elderly [17]. According to statistics from the American Osteoporosis Foundation (NOF) in 2018, between 1.5 and 2 million of the 10 million Americans currently were suffering from osteoporosis develop osteoporotic fractures each year [18]. 1/8 of men over the age of 50 have osteoporotic fractures. Thoracic vertebral compression fracture is a common type of osteoporotic fracture, which can cause a variety of complications, including back pain, chest tightness and hunchback, resulting in limited lung function. Compression fractures of the lumbar spine can cause bloating and abdominal pain, constipation, and loss of appetite. These illnesses make older people in relative financial difficulty more vulnerable to psychological symptoms, such as depression and loss of self-esteem [19, 20].

Osteoporosis has become a common disease in the middle-aged and elderly population. Its incidence has increased significantly. A more effective prevention and treatment measure is urgently needed to improve the clinical prognosis of such patients. Osteoporotic fractures will bring a heavy burden to society and economy. Clinical data have suggested that patients disabled by osteoporosis-related diseases have longer hospital stays than patients with other chronic diseases, which will lead to a dramatic increase in the medical costs of osteoporosis-related diseases [21]. Epidemiological data showed that in 2017, there were 3.24 million elderly patients with osteoporosis-related fractures in China, including 450,000 hip fractures, 1.31 million vertebral fractures, and 960,000 other osteoporotic fractures [22]. It is estimated that by 2050, there will be 5.99 million patients with osteoporotic fractures in China. According to the meta-analysis of Rizzoli, the overall prevalence of osteoporosis among people over 60 years old in my country is 36% (49% in women and 23% in men) [23].

Bushen Zhuanggu tablet is based on the theory of “kidney governing bone and marrow.” It is treated by nourishing the liver and kidneys, tonifying the qi and invigorating the blood, and forming prescriptions (*Eucommia ulmoides*, Herba Epimedii, Radix Scutellariae, Draconis, Radix *Angelicae sinensis*, *Codonopsis pilosula*, Radix Astragali, Dilong, etc.). At present, estrogen, calcium, bone formation enhancers, and bone resorption inhibitors are commonly used to treat PMOP. Although the targeted treatment of these drugs has significant clinical advantages, they pay too much attention to the local and ignore the overall concept, which is easy to cause complications of other systems [24]. The evidence showed that TCM could also effectively improve BMD, relieve bone pain and other symptoms. TCM has the advantages of rich resources, ideal efficacy, and little side effects, which provides a broad market for the treatment of PMOP [25]. The medicine is guided by the basic theory of Chinese medicine and combined with the clinical characteristics of osteoarthritis pain, clinical experience is constantly summarized and improved. In clinical practice, the medicine is mostly used for the back and leg pain caused by osteoporosis and osteoarthritis. However, its exact efficacy in postmenopausal osteoporosis treatment has not been revealed.

Our study demonstrated that in group A, the effective rate was 98.33%; in group B, the effective rate was 80.00%; and in group C,the treatment effective rate was 93.33%. The treatment effective rate of group A was the highest among different study groups. This suggested that no matter Bushen Zhuanggu tablet was used alone or Bushen Zhuanggu tablet was combined with conventional regimen, the clinical effect was more significant than that of conventional regimen. This is closely related to the prescription of Bushen Zhuanggu tablet. *Angelica sinensis* in the prescription can tonify the liver and kidney. Moreover, it can activate blood circulation and remove blood stasis. All kinds of medicines are combined, giving consideration to both exterior and interior, tonifying the kidney and filling essence, promoting blood circulation, promoting arthralgia, and dredging collaterals [26]. Bushen Zhuanggu tablet has a good curative effect in the treatment of PMOP, mainly because it can start from the etiology and pathology, improve the patient's condition, cure both the symptoms and the root causes, and have good short-term and long-term effects.

The results of this study showed that after 6 months of treatment, the levels of Ca, P, Scr, and PTH in the three groups decreased. The levels of Ca, P, Scr, and PTH in group A were lower than those in other groups. After intervention, the lumbar spine anteroposterior BMD, the left lateral femoral neck, and Ward's triangle bone mineral density were all increased in the three groups. Among them, group A was higher than B and C groups. After 6 months' treatment, the levels of PINP and OC in the three groups were increased, while the levels of *β*-CTX and ALP were decreased. BMD and bone quality indicates the bone strength. Others includes bone turnover, bone mineralization, and microfracture, in which bone turnover is the decisive factor of bone strength and can affect the formation of bone quality. On the other hand, the process of bone turnover is reflected by bone metabolic markers, which indirectly reflects osteoclasts activity. Bone metabolic markers are the products of the decomposition and synthesis of bone tissue itself, referred to as bone markers. BALP and *β*-CTX is the marker of bone formation and bone resorption, respectively. Bone metabolic markers can dynamically monitor the changes of bone formation and bone resorption after medication, which is helpful to judge the bone turnover rate and evaluate the curative effect [27, 28]. The improvement of various bone metabolism indexes in group A was significantly better than that in group B and C. This indicated that the adjuvant therapy of Bushen Zhuanggu tablet combined with conventional treatment could significantly improve the calcium and phosphorus metabolism and bone metabolism of the patients. The main reason is that the application of Bushen Zhuanggu tablet can improve the bone strength and bone quality of the patients.

The improvement effect of muscle strength in group A was significantly better than other groups. This showed that Bushen Zhuanggu tablet combined with routine treatment could significantly promote the limb function in patients with POMP. The main reason is that Bushen Zhuanggu tablet can improve patients' calcium and phosphorus metabolism, bone metabolism, BMD, and other physiological indexes. The improvement of these indexes is closely related to the improvement of muscle strength and the recovery of limb function, which will form a series of positive chain reactions. Modern medical research shows that there is a significant correlation between bone mass loss and muscle weakness [29, 30]. The improvement of muscle strength also contributes to the improvement of bone strength. The maximum load of weight-bearing bones after birth determines most of their strength. These loads come from muscle strength, so muscle strength can greatly affect the strength of our weight-bearing bones. When muscle exerts stress on bone, it will play a positive role in bone growth, remodeling, and maintenance of bone morphology to improve the strength of local bone under stress. Therefore, improving bone strength and increasing muscle strength is the key to reduce the fracture risk due to falls. The results illustrated that, the upper limb muscle strength of the three groups increased and TUGT shortened after 6 months of intervention. In addition, this study also found that there were significant differences in physiological function, life function, general health status, physical pain, mental state, emotional function, vitality, and social function scores among the three groups. The score of quality of life in group A was higher than that in B and C groups. Compared between groups, the incidence of fracture in group A was lower than that in group B and C at each time point. It is suggested that Bushen Zhuanggu tablet combined with conventional therapy can significantly improve the prognosis of patients with POMP and has a good preventive effect on the occurrence of fracture. The improvement in the quality of life of the patients is mainly due to the progressive improvement of their physical functions, their return to a normal life, their gradual integration into society, and a marked improvement in their physical and mental state. The decrease in the incidence of fracture is mainly due to the improvement of physiological indexes such as BMD, bone metabolism, and muscle strength, which can greatly reduce the risk of fracture. This study has some limitations; the sample size of this study is small, it belongs to a single-center study, and there is a certain deviation. There are patients' own factors and other confounding factors that may interfere with the accuracy of this study. In future research, we will carry out multicenter, large sample prospective studies, or we can draw more valuable conclusions.

To sum up, Bushen Zhuanggu tablet combined with conventional scheme is effective in the treatment of postmenopausal osteoporosis, which can significantly improve the BMD of patients, promote the recovery of limb function, and effectively prevent the occurrence of fracture. Bushen Zhuanggu tablet combined with conventional scheme is worthy of clinical promotion.

## Figures and Tables

**Figure 1:** The therapeutic effects among different groups.

**Figure 2:** Comparison of new bone fracture rate among different groups.

**Table 1:** Calcium and phosphorus metabolism indexes in three groups of patients [$\bar{x}\pm s$].

Group	*N*	Ca (mmol/L)		P (*μ*mol/L)		Scr (mmol/L)		PTH (pg/mL)	
		Before treatment	Treatment for 6 months	Before treatment	Treatment for 6 months	Before treatment	Treatment for 6 months	Before treatment	Treatment for 6 months
A group	60	2.08 ± 0.23	1.73 ± 0.36^a^	2.73 ± 0.56	1.98 ± 0.14^a^	94.23 ± 24.67	78.32 ± 13.02^a^	521.83 ± 57.08	435.08 ± 45.26^a^
B group	60	1.98 ± 0.31	2.06 ± 0.46	2.57 ± 0.39	2.41 ± 0.18	94.06 ± 25.02	90.29 ± 12.68^c^	518.32 ± 48.67	488.93 ± 41.47^c^
C group	60	2.03 ± 0.27	1.87 ± 0.38^b^	2.61 ± 0.48	2.25 ± 0.17^b^	93.87 ± 23.28	84.51 ± 15.13^b^	506.21 ± 53.72	477.92 ± 46.35^b^
*F*		2.028	10.169	1.793	105.093	0.003	11.534	1.420	24.624
*P*		>0.05	<0.05	>0.05	<0.05	>0.05	<0.05	>0.05	<0.05

Note: the comparison of group A, B, and C (*P* < 0.05) before and after treatment.

**Table 2:** Bone mineral density in three groups [$\bar{x}\pm s$, g/cm^2^].

Group	*N*	Lumbar vertebra orthopedic position(L_1_~L_4_)		Neck of left lateral femur		Ward's triangle area	
		Before treatment	Treatment for 6 months	Before treatment	Treatment for 6 months	Before treatment	Treatment for 6 months
A group	60	0.71 ± 0.23	0.92 ± 0.12^a^	0.63 ± 0.14	0.82 ± 0.07^a^	0.76 ± 0.18	0.89 ± 0.11^a^
B group	60	0.72 ± 0.21	0.77 ± 0.09	0.61 ± 0.18	0.64 ± 0.05	0.69 ± 0.17	0.71 ± 0.12
C group	60	0.69 ± 0.18	0.87 ± 0.16^c^	0.59 ± 0.15	0.71 ± 0.08^c^	0.72 ± 0.21	0.78 ± 0.08
*F*		0.325	21.830	0.966	107.391	2.106	45.046
*P*		>0.05	<0.05	>0.05	<0.05	>0.05	<0.05

Note: the comparison of group A, B, and C (*P* < 0.05) before and after treatment.

**Table 3:** Bone metabolic indexes between the two groups [$\bar{x}\pm s$].

Group	*N*	PINP (ng/mL)		*β*-CTX (ng/mL)		ALP (U/L)		OC (ng/mL)	
		Before treatment	Treatment for 6 months	Before treatment	Treatment for 6 months	Before treatment	Treatment for 6 months	Before treatment	Treatment for 6 months
A group	60	43.95 ± 11.63	61.47 ± 12.26^a^	0.66 ± 0.13	0.43 ± 0.08^a^	99.41 ± 12.88	71.62 ± 12.08^a^	5.62 ± 1.03	9.87 ± 1.83^a^
B group	60	45.02 ± 11.71	48.72 ± 13.04	0.62 ± 0.11	0.59 ± 0.03^b^	99.21 ± 12.67	86.54 ± 12.51^b^	5.72 ± 1.13	6.05 ± 1.22
C group	60	44.71 ± 12.08	54.33 ± 11.48^c^	0.61 ± 0.14	0.52 ± 0.06^c^	98.56 ± 13.34	76.63 ± 11.71^c^	5.34 ± 1.18	7.26 ± 1.47^c^
*F*		0.130	10.838	16.257	106.239	0.070	23.609	1.872	98.033
*P*		>0.05	<0.05	>0.05	<0.05	>0.05	<0.05	>0.05	<0.05

Note: the comparison of group A, B, and C (*P* < 0.05) before and after treatment.

**Table 4:** Upper limb muscle strength and TUGT between the two groups [$\bar{x}\pm s$].

Group		*N*	Upper body strength (kg)		TUGT (s)	
			Before treatment	Treatment for 6 months	Before treatment	Treatment for 6 months
A group		60	18.32 ± 2.47	27.64 ± 1.13^a^	10.45 ± 1.46	7.44 ± 1.03^a^
B group		60	18.11 ± 2.82	20.06 ± 1.15^b^	10.66 ± 1.42	9.04 ± 1.26^b^
C group		60	17.74 ± 3.05	22.34 ± 1.14^c^	10.52 ± 1.29	8.57 ± 1.14^c^
*F*			0.665	698.216	0.354	30.836
*P*			>0.05	<0.05	>0.05	<0.05

Note: the comparison of group A, B, and C(*P* < 0.05) before and after treatment.

**Table 5:** Quality of life scores among the three groups before treatment ($\bar{x}\pm s$, points).

Group	*N*	Physiological function	Physiological function	Somatic pain	General state of health	Mentality	Social function	Emotional function	Vitality
A group	60	61.12 ± 5.22	62.25 ± 5.36	61.47 ± 5.27	62.23 ± 5.10	61.17 ± 4.49	61.15 ± 4.48	60.88 ± 4.50	60.28 ± 5.77
B group	60	61.38 ± 5.37	62.31 ± 5.44	61.12 ± 5.10	62.98 ± 5.24	61.08 ± 4.42	61.09 ± 4.45	60.22 ± 4.45	61.03 ± 5.63
C group	60	61.00 ± 5.20	62.98 ± 5.60	60.99 ± 5.18	62.04 ± 5.02	61.01 ± 4.39	60.89 ± 4.42	60.34 ± 4.69	60.86 ± 5.60
*F*		0.082	0.330	0.138	0.565	0.007	0.056	0.359	0.289
*P*		>0.05	>0.05	>0.05	>0.05	>0.05	>0.05	>0.05	>0.05

**Table 6:** Quality of life scores among the three groups after treatment ($\bar{x}\pm s$, points).

Group	*N*	Physiological function	Physiological function	Somatic pain	General state of health	Mentality	Social function	Emotional function	Vitality
A group	60	77.38 ± 5.41^a^	76.42 ± 6.01^a^	76.23 ± 6.18^a^	75.98 ± 4.63^a^	73.82 ± 5.41^a^	78.89 ± 4.62^a^	81.56 ± 3.47^a^	71.16 ± 5.42^a^
B group	60	68.46 ± 4.87^b^	63.41 ± 5.62^b^	66.71 ± 6.02^b^	65.32 ± 5.12^b^	64.45 ± 5.61^b^	70.03 ± 3.87^b^	73.23 ± 3.15^b^	64.28 ± 4.72^b^
C group	60	72.25 ± 5.02^c^	71.89 ± 5.37^c^	72.01 ± 5.07^c^	71.29 ± 5.07^c^	70.02 ± 5.16^c^	75.42 ± 4.26^c^	78.55 ± 3.37^c^	67.81 ± 5.24^c^
*F*		46.139	81.320	40.902	70.044	45.760	65.868	96.114	26.903
*P*		<0.05	<0.05	<0.05	<0.05	<0.05	<0.05	<0.05	<0.05

Note: the comparison of group A, B, and C (*P* < 0.05) before and after treatment.

## Data Availability

The datasets used and analyzed during the current study are available from the corresponding author upon reasonable request.
